# Alpha-Glucosidase Inhibitory Assay-Screened Isolation and Molecular Docking Model from *Bauhinia pulla* Active Compounds

**DOI:** 10.3390/molecules26195970

**Published:** 2021-10-01

**Authors:** Sukanya Dej-adisai, Ichwan Ridwan Rais, Chatchai Wattanapiromsakul, Thanet Pitakbut

**Affiliations:** 1 Department of Pharmacognosy and Pharmaceutical Botany, Faculty of Pharmaceutical Sciences, Prince of Songkla University, Hat Yai 90112, Songkhla, Thailand; ichwan.rais@pharm.uad.ac.id (I.R.R.); chatchai.w@psu.ac.th (C.W.); 2 Department of Pharmaceutical Biology, Faculty of Pharmacy, Universitas Ahmad Dahlan, Yogyakarta 55164, Indonesia; 3 Department of Biochemical and Chemical Engineering, Technical University of Dortmund, 44227 Dortmund, Germany; thn_ptb@hotmail.com

**Keywords:** *Bauhinia pulla*, anti-diabetic, alpha-glucosidase inhibition, molecular docking

## Abstract

The aim of this research was to establish the constituents of *Bauhinia pulla* as anti-diabetic agents. A phytochemistry analysis was conducted by chromatographic and spectroscopic techniques. The alpha-glucosidase inhibitory assay screening resulted in the isolation of eight known compounds of quercetin, quercitrin, luteolin, 5-deoxyluteolin, 4-methyl ether isoliquiritigenin, 3,2′,4′-trihydroxy-4-methoxychalcone, stigmasterol and β-sitosterol. Ethanol leaf extracts showed potential effects, which led to a strong inhibitory activity of isolated quercetin at 138.95 µg/mL and 5.41 µg/mL of IC_50_, respectively. The docking confirmed that flavonoids and chalcones had the same potential binding sites and responsibilities for their activity. This study was the first report of *Bauhinia pulla* chemical constituents and its alpha-glucosidase inhibition.

## 1. Introduction

The amount of the population with diabetes has escalated significantly in the last two decades and exhibits it as a global epidemic malady [1]. One diabetes therapy management approach is alpha-glucosidase inhibitor medication development. Alpha-glucosidase inhibitors (such as acarbose) slow the digestion of carbohydrates by reversible and competitive inhibition. The postprandial glucose rise in the blood is dose-related and, therefore, decreased due to the down-regulation of direct glucose absorption [2]. Thus, alpha-glucosidase inhibitors are becoming a notable strategy for treating type 2 diabetes. The interaction between the alpha-glucosidase enzyme and its inhibitors is still interesting to investigate. The binding mechanism of the alpha-glucosidase inhibitor is important and could present beneficial evidence by molecular docking [3]. Despite its potential, acarbose has been found to cause gastrointestinal discomforts such as flatulence and diarrhea [4]. Wongon and Limpeanchob (2020) reported that acarbose and other alpha-glucosidase inhibitors cause gastrointestinal discomfort (flatulence and diarrhea) due to the rising fermentation of undigested polysaccharides by bacteria living in the intestine and generating intestinal gas production [5]. Some plants from the *Bauhinia* genus have shown promising antibacterial activities, as reported by Cechinel-Zanchett et al. [6]. Therefore, using *Bauhinia pulla* as an anti-glucosidase agent may prevent side effects caused by acarbose and other alpha-glucosidase inhibitors.

Herbal remedies are important in the medication system, placing herbal medicines as interesting low-cost alternatives. Therefore, it is important to increase their quality and potency. Concomitantly, finding new potential compounds fuels recent drug development research, leading the way in compound bio-assay modeling [7]. Previously, Fabaceae plants have exhibited potential alpha-glucosidase inhibition. The *Bauhinia* genus, in the Fabaceae family, has performed with higher activity than acarbose [8]. *Bauhinia* is widely spread in Thailand, with approximately twenty-five species identified in northeast Thailand [9]. *Bauhinia* is reported to contain flavonoids, phenolics, and terpenoids, which are responsible for their activity. Commonly, these secondary metabolite groups have mainly played an important role as potential phytomedicines. They were discovered and studied as diabetic treatments from plants. Further, these groups were more suitable as a chemical model on anti-diabetic phytopreparation profiling [10].

*Bauhinia pulla,* as one of the Fabaceae plants in Thailand, is traditionally used as a treatment for menstrual disorders and blood tonic [11]. The bark and sapwood exhibited cytoprotective activity against glutamate-induced cell damage and degeneration in HT22 cells [12]. Based on a preliminary assay on alpha-glucosidase inhibition, *Bauhinia pulla* showed potential inhibitory activity. However, this plant has not been reported in phytochemical investigations or alpha-glucosidase inhibitory activities. Therefore, the present study was to conduct new additional phytochemical information from *Bauhinia pulla* and its activity as an alpha-glucosidase inhibitory agent.

## 2. Results and Discussion

### 2.1. Fractionation and Isolation Screening Based on Bioactivity

Screening on alpha-glucosidase inhibitory activity was used to classify the active extracts from *Bauhinia pulla*, as shown in Table 1. The screening results showed that all extracts exhibited more than 50% alpha-glucosidase inhibition, except for the n-hexane extract. The ethanol leaves extract (ETLBP) showed the potential inhibitory effect, with a 138.95 µg/mL IC_50_ value, a mild value, lower than the standard acarbose value of 193.37 µg/mL. Further, the study continued to investigate natural compounds responsible for this effect.

### 2.2. Identification of the Isolated Compounds

The isolated compounds were identified by their ^1^H- and ^13^C-NMR, FT-IR, and MS, as well as by comparison of reported spectral data in the literature. The isolated compounds from *Bauhinia pulla* were two mixed compounds and six pure compounds. Two mixed compounds were known as the mixture of stigmasterol (**1a**) and β-sitosterol (**1b**); the mixture of stigmasterol (**2a**) and β-sitosterol glycoside (**2b**). Six pure compounds were known as quercetin (**3**); quercitrin (**4**); luteolin (**5**); 5-deoxyluteolin (**6**); 4-methyl ether isoliquiritigenin (**7**); 3,2’,4’-trihydroxy-4-methoxychalcone (**8**). The chemical structures of *Bauhinia pulla* isolated compounds one to eight are shown in Figure 1.

The mixture of stigmasterol and β-sitosterol (**1a**, **1b**): white amorphous powder (CHCl_3_); UV λ_max_ (CHCl_3_) nm: 290; IR cm^−l^: 3630, 3368, 3017, 2943, 2834, 1631, 1216, 1027; C_29_H_48_O:C_29_H_50_O; ^1^H NMR (CDCl_3_) δ: 5.01 (1 H, dd, J = 15.0, 8.5 Hz) and 5.13 (1 H, dd, J = 15.0, 8.5 Hz) were assigned as H-22 and H-23 of stigmasterol, respectively. The δ 5.33 (1H, brd, J = 5.0 Hz) was assigned as H-6 of both b-sitosterol and stigmasterol [13]. Complete data were not shown. The integration of H-6, H-22 and H-23 were in the ratio of 1.00:0.26:0.27.

The mixture of stigmasterol and β-sitosterol glycoside (**2a**, **2b**): white amorphous powder (CHCl_3_:MeOH); UV λ_max_ (CHCl_3_:MeOH) nm: 290; IR cm^−l^: 3433, 2954, 2930, 2849, 1642, 1455, 1378, 1016; C_29_H_48_O:C_29_H_50_O and 2C_6_H_12_O_6_; ^1^H NMR data were identical to the mixture of stigmasterol and β-sitosterol when compared with previously reported values [14]. The sugar spectrum appeared in the δ range 3.20–4.40 ppm.

Quercetin (**3**): yellow powder (MeOH); UV λ_max_ (MeOH) nm: 370; IR cm^−l^: 3407, 1664, 1521, 1262, 1092, 1014, 783; C_15_H_10_O_7_; MS m/z: 302.04 ([M+Na]^+^); ^l^H NMR (CD_3_OD) δ: 7.72 (lH, d, J = 2.0 Hz, H-2’), 7.62 (lH, dd, J = 8.5, 2.0 Hz, H-6’), 6.85 (lH, d, J = 8.0 Hz, H-5’), 6.37 (lH, d, J = 2.0 Hz, H-8), 6.16 (lH, d, J = 2.0 Hz, H-6). The ^l^H NMR spectrum was compared with prior studies [15].

Quercitrin (**4**): yellow powder (MeOH); UV λ_max_ (MeOH) nm: 285, 350; IR cm^−l^: 3391, 1656m, 1608, 1449, 1202, 1060, 879,), 2933-2852 (sugar); C_21_H_20_O_11_; MS m/z: 448.1 ([M+Na]^+^); ^l^H NMR (CD_3_OD) δ: 7.33 (lH, d, J = 2.2 Hz, H-2’), 7.29 (lH, dd, J = 8.3, 2.2 Hz, H-6’), 6.91 (lH, d, J = 8.2 Hz, H-5’), 6.36 (lH, d, J = 2.0 Hz, H-8), 6.19 (lH, d, J = 2.0 Hz, H-6). Proton of sugar moieties δ: 5.34 (lH, d, J = 1.5 Hz, H-1’’), 4.21 (lH, dd, J = 3.4, 1.7 Hz, H-2’’), 3.75 (lH, dd, J = 9.3, 3.4 Hz, H-3’’), 3.42 (lH, dd, J = 9.5, 6.4 Hz, H-5’’), 3.34 (lH, d, J = 9.5 Hz, H-4’’), 0.94 (3H, d, J = 6.1 Hz, H-6’’). The NMR spectra were based on a data comparison with a prior study [16].

Luteolin (**5**): yellow amorphous powder (MeOH); UV λ_max_ (MeOH) nm: 348; IR cm^−l^: 3400, 2948, 1654, 1450, 1113, 1023, 719; C_15_H_10_O_6_; MS m/z: 286.05 ([M+H]^+^); ^1^H NMR (CD_3_OD) δ: 7.38 (1H, dd, J = 8.8, 2.0 Hz, H-6’), 7.37 (1H, d, J = 2.2 Hz, H-2’), 6.90 (1H, d, J = 8.8 Hz, H-5’), 6.53 (1H, s, H-3), 6.43 (1H, d, J = 1.95 Hz, H-8), 6.20 (1H, d, J = 1.95 Hz, H-6). The NMR spectra were compared with a prior study [17].

5-deoxyluteolin (**6**): yellow amorphous powder (MeOH); UV λ_max_ (MeOH) nm: 365; IR cm^−l^: 3368, 2945, 1654, 1450, 1113, 1027, 672; C_15_H_9_O_5_; MS m/z: 270.05 ([M+Na]^+^); ^1^H NMR (CD_3_OD) δ: 7.60 (1H, d, J = 9.0 Hz, H-5), 7.51 (1H, d, J = 2.0 Hz, H-2’’), 7.23 (1H, dd, J = 8.5, 2.0 Hz, H-6’), 6.83 (1H, d, J = 8.5 Hz, H-5’), 6.69 (1H, s, H-3), 6.68 (1H, d, J = 2.5 Hz, H-8), 6.67 (1H, dd, J = 9.5, 2.0 Hz, H-6). The NMR spectra were compared with a prior study [18].

4-methyl ether isoliquiritigenin (**7**): yellow needles (MeOH); UV λ_max_ (MeOH) nm: 365; IR cm^−l^: 3430, 2846, 1631, 1605, 1458, 1033, 976; C_16_H_14_O_4_; MS m/z: 270.09 ([M+H]^+^); ^1^H NMR (CD_3_OD) δ: 7.97 (1H, d, J = 9.0 Hz, H-6’), 7.81 (1H, d, J = 15.3 Hz, H-β), 7.70 (2H, d, J = 6.8 Hz, H-2, 6), 7.63 (1H, d, J = 15.3 Hz, H-α), 6.98 (2H, d, J = 6.8 Hz, H-3, 5), 6.42 (1H, dd, J = 8.7, 2.4 Hz, H-5’), 6.29 (1H, d, J = 2.4 Hz, H-3’), 3.81 (3H, s, -OCH_3_). ^13^C NMR (CD_3_OD) δ: 193.5 (C=O), 167.6 (C-4’, s), 166.5 (C-2’, s), 163.4 (C-4, s), 145.2 (C-β, s), 133.4 (C-6’, s), 131.6 (C-2, 6, d), 129.0 (C-1, s), 119.3 (C-α, s), 115.5 (C-3, 5, d), 114.7 (C-1’, s), 109.2 (C-5’, s), 103.8 (C-3’, s). The NMR spectra were compared with a prior study [17].

3,2’,4’-trihydroxy-4-methoxychalcone (**8**): yellow amorphous powder (MeOH); UV λ_max_ (MeOH) nm: 300, 370; IR cm^−l^: 3368, 2946, 2834, 1654, 1450, 1027; C_16_H_14_O_5_; ^1^H NMR (CD_3_OD) δ: 7.96 (1H, d, J = 9.0 Hz, H-6’), 7.74 (1H, d, J = 16.0 Hz, H-β), 7.60 (1H, d, J = 15.5 Hz, H-α), 7.23 (1H, d, J = 2.0 Hz, H-2), 7.20 (1H, dd, J = 8.5, 2.0 Hz, H-6), 6.98 (1H, d, J = 8.5 Hz, H-5), 6.42 (1H, dd, J = 9.0, 2.5 Hz, H-5’), 6.28 (1H, d, J = 2.5 Hz, H-3’), 3.90 (3H, s, -OCH_3_). The NMR spectra were compared with a prior study [19].

### 2.3. Alpha-Glucosidase Inhibitory Assay

As shown in Table 2, we divided the compounds into two groups based on the IC_50_ values. Group-one, with quercetin (IC_50_ = 5.41 µg/mL) and quercitrin (IC_50_ = 49.69 µg/mL) showed potential inhibitory activity stronger than acarbose. Their IC_50_ values were 22.9 and 2.5 times lower than acarbose, respectively. Group-two, including another three flavonoids, two chalcones, and two mixed-steroids, exhibited moderate to weak inhibitory activity. The inhibitory effect of compounds against alpha-glucosidase activity depended on the pharmacophore and its structural modification. Despite the inhibitory potency, in this study, anti-alpha-glucosidase activity from 3,2’,4’-trihydroxy-4-methoxychalcone was reported for the first time. Unlike flavonoids, our understanding regarding how chalcone derivatives inhibited glucosidase activity is still limited. Up to date, Rocha et al. (2019) is the most comprehensive and recent study investigating anti-glucosidase activity from chalcone derivatives, but only 41 compounds were studied. In Rocha’s study, the hydroxy group was shown a favor inhibitory activity and concluded that more hydroxy groups contributed to the stronger activity [20]. However, our obtained result indicated differently. As presented in Figure 1, the only chemical variant between 4-methyl ether isoliquiritigenin (compound 7) and 3,2’,4’-trihydroxy-4-methoxychalcone (compound 8) was a hydroxy group at ring B position (benzylidene). However, the activity of 3,2’,4’-trihydroxy-4-methoxychalcone was lower than 4-methyl ether isoliquiritigenin by approximately 6-fold even 3,2’,4’-trihydroxy-4-methoxychalcone had more hydroxy group than 4-methyl ether isoliquiritigenin (Table 2). Despite the similarity between flavonoids and chalcones, adding a more hydroxy group in the flavonoid structure improved the inhibitory activity by nearly four times, comparing the IC_50_ values between luteolin (compound 5) and 5-deoxyluteolin (compound 6). Interestingly, a similar behavior was observed when the sugar moiety was added into flavonoid and steroid structures, even though both natural product classes did not relate. In both cases, the inhibitory activity was dropped by roughly 10-fold, compared with quercetin (compound 3) and quercitrin (compound 4), and by nearly 6-fold compared with a mixture of steroids (compound 1) and a mixture of steroid glycosides (compound 2), as shown in Table 2.

### 2.4. Computerized Molecular Docking

The first and most important step in performing molecular docking is to validate the docking protocol. As Morris et al. (2009) [21] suggested, validating the established docking protocol before experimenting is essential. The acceptance criterion is that the RMSD of the re-docked native ligand and its original pose should be less than 3.5 Å. Our validation result exhibited an RMSD of less than 1 Å. Therefore, our protocol passed this criterion.

As shown in Figure 2A, our molecular docking revealed that both flavonoids and chalcones from *Bauhinia pulla* could insert themselves into the active site of the glucosidase. The finding here was expected since chalcone is a flavonoid precursor, their structural similarities may lead them to have the same binding site, which was in good agreement with the previous studies from both flavonoids and chalcones. Therefore, our docking results were in line with earlier studies [22,23].

The molecular docking has shown that two isolated chalcones from *Bauhinia pulla*, 4-methyl ether isoliquiritigenin and 3,2’,4’-trihydroxy-4-methoxychalcone, had a similar structural alignment in the binding pocket of glucosidase, as presented in Figure 2B. Both chalcones inserted in the ring B position (benzylidene) deep inside the pocket at the same binding site as glucose, a natural substrate, while the ring A position (acetophenone) laid at the entry site of the pocket (Figure 2B). Noticeably, the 2D diagrams indicated that two chalcones interacted with Asp 352, acting as a transitional state stabilizer (one of the catalytic residues), as depicted in Figure 2C,D. However, only 4-methyl ether isoliquiritigenin was able to bind with Asp 215, acting as a nucleophile (the other catalytic residues) as shown in Figure 2D [24]. Interestingly, they also bound with neighboring amino acids in the active site, including Asp 69 and His 112. However, only 3,2’,4’-trihydroxy-4-methoxychalcone formed a hydrogen bond with an amino acid at the entrance, Tyr 158, as shown in Figure 2D [25]. As mentioned earlier, a recent study on the structure-activity relationship (SAR) between chalcones and glucosidase reported that the hydroxy substitution on chalcone played an essential role in the inhibitory activity against glucosidase, but the methoxy substitution did not favor this activity [20]. However, our in vitro experiment did not agree with the previous report and showed that 4-methyl ether isoliquiritigenin with two hydroxyl substitutions had better inhibitory activity than 3,2’ 4’-trihydroxy-4-methoxychalcone with three hydroxyl substitutions (Table 2). Therefore, we performed a rescoring simulation from our docking poses using Autodock 4.2.6 to understand better the impact of the chalcone properties involving the molecular interaction. The rescoring revealed that an extra hydroxyl substitution in 3,2’,4’-trihydroxy-4-methoxychalcone only slightly improved the binding energy by 0.10 kcal/mol compared to 4-methyl ether isoliquiritigenin based on the simulation. However, the rescoring still indicated a positive relationship between the hydroxyl group and the glucosidase inhibitory activity. After carefully evaluating each parameter in the rescoring simulation, we found that two parameters, such as electrostatic and torsional free energies from 4-methyl ether isoliquiritigenin, were lower than 3,2’,4’-trihydroxy-4-methoxychalcone (Table 3). These two parameters might explain why 4-methyl ether isoliquiritigenin showed better inhibitory activity than 3,2’,4’-trihydroxy-4-methoxychalcone and both linked with an extra hydroxy group. Recently, Lu et al. [26] reported that more hydroxyl groups contributed to higher electrostatic energy. Therefore, Lu’s study supported our finding from the rescoring simulation, explaining lower electrostatic energy from 4-methyl ether isoliquiritigenin due to less hydroxyl group than 3,2’ 4’-trihydroxy-4-methoxychalcone [26]. However, electrostatic energy might not have a significant impact since the difference between the two chalcones was small. On the other hand, Hadni and Elhallaoui (2019) reported an impact of torsion energy in antimalarial activity. In their study, a molecule with more torsion energy showed less activity [27]. Therefore, lower torsion energy contributed to a better activity, which agreed with our rescoring simulation and in vitro assay of 4-methyl ether isoliquiritigenin and 3,2’ 4’-trihydroxy-4-methoxychalcone earlier.

Our molecular docking and rescoring simulation proposed a novel possible explanation regarding the negative effect of the hydroxy group on the chemical structure of chalcone, and this new finding was not mentioned in the previous report from Rocha et al. [20]. Therefore, we are hereby presenting a new piece of evidence and purposing a negative impact of the hydroxy substitution at ring B on the chalcone structure that decreases the anti-glucosidase activity based on our molecular docking and rescoring simulations.

For flavonoids, our molecular docking experiment showed that all four flavonoids could interact with the Asp 215/ Glu 277/ Asp 352 triangles (Figure 2E,J). These triangles were responsible for the catalytic reaction of the glucosidase, and binding with one of these residues could inhibit the glucosidase hydrolysis activity. Thereby, our results here indeed support the earlier findings of flavonoids and their inhibitory activity against glucosidase [22,23].

## 3. Discussion

From the flavonoid chemical structure, the intended effect was given by OH group number and position as the determinant factor. Quercetin was the most active because it has hydroxylation at a critical position for the alpha-glucosidase inhibition of flavonoids which are 5, 7, or 8-positions of ring A; at 3’ and 4’-positions of ring B; and 3-position of ring C, as well as the double bond of C2=C3 in ring C [23]. This explanation showed the relationship between the structure configuration with the inhibitory activity of quercetin. It performed a strong inhibitory effect 22.9-fold lower than the acarbose. According to a previous study, quercetin exhibited alpha-glucosidase inhibitory activity at IC_50_ = 15 µM [23], slightly lower than the present result with IC_50_ = 5.41 µg/mL (20 µM). Thus, this study provided additional information that quercetin was responsible for *Bauhinia pulla* activity as an alpha-glucosidase inhibitor.

It is currently accepted that hydroxy group modification or elimination in flavonoids will reduce the alpha-glucosidase inhibitory effects of flavonoids [23]. Therefore, quercitrin with rhamnose replacement on the 3-position of ring C and luteolin with hydroxy elimination on the 3-position of ring C had higher IC_50_ values than quercetin. Moreover, 5-deoxyluteolin with hydroxy elimination on the 5-position of ring A was 3.5-fold higher compared to luteolin. In contrast with chalcones, the presence of a hydroxy group on the 3- or 5-positions of ring B of 3,2’,4’-trihydroxy-4-methoxychalcone reduced the activity and was 5.8 times higher compared to 4-methyl ether isoliquiritigenin. In terms of sugar presence in flavonoid and steroid structures, the inhibitory activity was lower, as mentioned above.

Flavonoids and chalcones are common secondary metabolites that are found together in many medicinal plants, especially from the Fabaceae family, since chalcones are the precursor of flavonoids [28,29]. Moreover, these two groups of secondary metabolites usually exhibit the same trend in bioactivities from anti-oxidant to anti-cancer effects [30]. However, it seems that only flavonoids were thoroughly investigated on the anti-glucosidase activity [23] when compared to its precursors, chalcones. Therefore, to fill the gap of knowledge, molecular docking was performed to evaluate the molecular interaction between flavonoids, chalcones and alpha-glucosidase.

Molecular interaction between the ligand of interest and target protein could be evaluated by applying sophisticated computational techniques, also known as molecular docking. This approach has been used to examine and visualize a possible molecular interaction of the ligand-protein complex. Therefore, we applied this technique in this study to provide a better understanding of the molecular interaction of flavonoids, chalcones and glucosidase.

From the discussion earlier, flavonoids and chalcones were known as alpha-glucosidase inhibitors, where substitution of the hydroxyl group may reduce the inhibitory effects. Molecular docking was used to confirm the activity, which revealed the same binding site between flavonoids and chalcones from *Bauhinia pulla*. This also provided new evidence showing the negative impact of the hydroxy substitution at ring B on the chalcone structures, contributing to higher electrostatic and torsion energies (less stability). This new information could explain the potency of the glucosidase inhibitory activity of chalcone and benefit for the further drug design of its derivatives.

## 4. Materials and Methods

### 4.1. General

IR spectra of isolated compounds were measured by Perkin Elmer FT-IR Spectrum One Spectrometer. NMR spectra were obtained by Fourier Transform NMR Spectrometer (^1^H-NMR 500 MHz and ^13^C-NMR 125 MHz), model UNITY INNOVA, Varian. Electron spray ionization mode (ESI) of MS was observed on Alliance-micromass Waters 2690-LCT

### 4.2. Plant Extract Preparation

The leaves and wood of *Bauhinia pulla* (BP) were collected from the Central Thai Literary Botanical Garden, Ratchaburi, Thailand, in January 2017. *Bauhinia pulla* was identified by taxonomist Ms. Pranee Rattanasuwan and kept as a herbarium specimen (SKP 072 02 23 01) at the Department of Pharmacognosy and Pharmaceutical Botany, Faculty of Pharmaceutical Sciences, Prince of Songkla University, Songkhla Province, Thailand. *Bauhinia pulla* leaves (L) and wood (W) were washed and dried at 50 ºC in a hot air oven for 24 h and powdered by a grinder.

The dried leaves (3.31 kg) and wood (6.80 kg) powder were extracted separately with 10 L of *n*-hexane (H) at room temperature for three days and re-macerated three times. Solvent evaporation yielded a crude extract named HLBP (36.31 g). The marc was then re-extracted by successive solvent maceration with 10 L of ethyl acetate (EA), ethanol (ET) and boiled water (W) to obtain EALBP (87.08 g), ETLBP (414.80 g), WLBP (273.45 g) from the leaves; HWBP (8.57 g), EAWBP (17.15 g), ETWBP (630.73 g), WWBP (234 g) from the wood.

### 4.3. Alpha-Glucosidase Inhibitory Assay

Acarbose and other chemicals of the alpha-glucosidase inhibitor assay were purchased from Sigma-Aldrich (St. Louis, MO, USA). The assay protocol was performed as reported previously [8], enzymatic degradation of substrate *p*-nitrophenyl-D- glucopyranoside (*p*NPG) by glucosidase enzyme was observed as *p*-nitrophenol (*p*NP), a yellow product which absorbed at 405 nm of UV light every 30 s for 5 min in a microplate reader. Briefly, the enzyme from *Saccharomyces cerevisiae* (EC 3.2.1.20) and the *p*NPG substrate were dissolved in 0.1 M phosphate buffer (pH 7), which was enriched by bovine serum albumin and sodium azide. Standards and samples were suspended in 20% (*v*/*v*) of DMSO in a water solution. In a 96-well plate, 50 µl of PBS, standards, samples and enzyme solutions were mixed and incubated for 2 min at 37 °C. At last, 50 µl of 4 mM *p*NPG was added and incubated for 5 min before the kinetic parameter measurement, as described earlier.

The velocity was examined by a linear relationship equation between absorbance and time, Equation (1).

Velocity = (∆ Absorbance at 405 nm)/(∆ Time)(1)

The percent inhibition was determined for the highest velocity as:

% Inhibition = (V control − V sample)/(V control) × 100(2)

The IC_50_ value was calculated by using a calibration curve equation between samples at five different concentrations and inhibition percentages.

### 4.4. Bioassay-Guidance Isolation

Eight solvent extracts from the leaves and wood of *Bauhinia pulla* were screened by alpha-glucosidase inhibitory assay to evaluate the potential active extract. The result of alpha-glucosidase inhibition from each extract was used for guidance in the bioactive compounds isolation process. Compounds were isolated by chromatographic methods such as thin-layer, column and size-exclusion chromatography. Compounds were interpreted by spectroscopic methods such as ^1^H-NMR, ^13^C-NMR and high-resolution mass spectrometry.

The fractions resulting from the quick column were then isolated by classical column chromatography by using variable mixtures of *n*-hexane and ethyl acetate, *n*-hexane and chloroform, chloroform and methanol. The last step of purification was isolated by gel filtration column chromatography (Sephadex^®^) with the mobile phase of absolute methanol or 10% chloroform in methanol.

### 4.5. Computerized Molecular Docking

Alpha-glucosidase of *S. cerevisiae* (PDB ID: 3A4A) from the NCBI PDB database (https://www.rcsb.org accessed on 12 August 2021) was chosen as the target protein, whereas the compounds of interest were searched through the PubChem database (https://pubchem.ncbi.nlm.nih.gov accessed on 12 August 2021) and downloaded. For molecular docking, Autodock Vina version 1.1.2, developed by the Scripps Research Institute, San Diego, CA, USA, was used to examine the molecular interaction [31]. The glucosidase was carefully prepared for docking, and the active site was located before performing the molecular docking by Autodock Tool version 1.5.6. The native glucose molecule was used as a navigator to find the binding pocket [32]. The coordination of the pocket was set up at the center of X = 21.5, Y = −7.4 and Z = 24.1, respectively and the size of the pocket was adjusted as a cubic box, which had the size of 16 Å × 16 Å × 16 Å. On the other hand, the selected compounds were properly prepared by Avogadro Version 1.2.0, in which two optimization steps were applied both geometrically and energetically [33]. The merck molecular force field (MMFF) 94 force field was applied for energy optimization [34]. To perform the molecular docking, almost all of the parameters were set to default, except the exhaustiveness, which was adjusted to 24. For the post docking analysis, the Viewdock package from Chimera, version 1.11.2, was selected for the visualization [35] and discovery; the studio visualizer free version (20.1.0.19295) was used to generate the interaction diagram [36]. A rescoring simulation was performed by using the Autodock4 version 4.2.6 following our previous report [21,37].

## 5. Conclusions

Eight compounds were isolated from *Bauhinia pulla* containing flavonoids, chalcones and the mixture of steroid and steroidal glycoside. *Bauhinia pulla* ethanol leaf extract, and its isolated quercetin, showed the highest alpha-glucosidase inhibition. Molecular docking was used to confirm that flavonoids and chalcones from *Bauhinia pulla* had the same binding site in the models as the potential group compounds and are responsible for the activity of alpha-glucosidase inhibition. This study was the first report of *Bauhinia pulla* chemical constituents and their anti-diabetic activity via alpha-glucosidase inhibition. This published manuscript is based on the Ph.D. thesis of co-author Ichwan Ridwan Rais [38].

## Figures and Tables

**Figure 1:** The chemical structure of *Bauhinia pulla* isolated compounds.

**Figure 2:** The molecular interaction between amino acids in the active site of glucosidase (Ivory) and glucose as a native ligand (White) and isolated flavonoids, luteolin (Blue), 5-deoxyluteolin (Pink), quercetin (Green), quercitrin (Yellow), chalcones, 3,2’,4’-trihydroxy-4-methoxychalcone (Red) and 4-methyl ether isoliquiritigenin (Cyan) from *Bauhinia pulla* (**A**). Structural alignment of 3,2’,4’-trihydroxy-4-methoxychalcone (Red) and 4-methyl ether isoliquiritigenin (Cyan) in the active site of glucosidase (Ivory) (**B**). 2D interaction diagram of 4-methyl ether isoliquiritigenin-glucosidase complex (**C**), 3,2’,4’-trihydroxy-4-methoxychalcone-glucosidase complex (**D**), quercetin-glucosidase complex (**E**), quercitrin-glucosidase complex (**F**), luteolin-glucosidase complex (**I**), and 5-deoxyluteolin-glucosidase complex (**J**). Catalytic residues in the active site indicated by red boxes and asterisks. A, B and C indicate the ring system in both flavonoids and chalcones.

**Table 1:** Alpha-glucosidase inhibition test for *Bauhinia pulla* extract screening.

Part	Extract	Alpha-Glucosidase Inhibition (%) ± SD	IC_50_ (µg/mL)
**Leaves**	*n*-Hexane (HLBP)	15.09 ± 3.09	-
	Ethyl acetate (EALBP)	52.34 ± 4.41	529.60
	Ethanol (ETLBP)	97.44 ± 0.92	138.95
	Water (WLBP)	54.08 ± 3.30	641.66
**Woods**	*n*-Hexane (HWBP)	29.36 ± 2.12	-
	Ethyl acetate (EAWBP)	58.73 ± 0.98	957.13
	Ethanol (ETWBP)	69.53 ± 2.29	693.98
	Water (WWBP)	58.59 ± 3.06	655.36
**Standard**	Acarbose	86.09 ± 1.54	193.37

**Table 2:** Alpha-glucosidase inhibition of isolated compounds from *Bauhinia pulla*.

Compounds	Extract	IC_50_ (µg/mL)	Proportion *
**Acarbose**	-	124.11	-
**Quercetin**	EALBP, ETLBP, ETWBP	5.41	22.94
**Quercitrin**	ETLBP	49.69	2.50
**Luteolin**	ETWBP	164.05	0.76
**5-deoxyluteolin**	ETWBP	574.57	0.22
**4-methyl ether isoliquiritigenin**	EAWBP, ETWBP	220.05	0.56
**3,2’** **,4’-trihydroxy-4-methoxychalcone**	ETWBP	1273.31	0.10
**Steroids**	EALBP, HWBP, ETWBP	1392.81	0.09
**Steroids glycoside**	ETLBP	8204.20	0.02

* IC50 of each isolated compound was compared with standard acarbose.

**Table 3:** Rescoring of the selected docking poses of 4-methyl ether isoliquiritigenin (compound 7) and 3,2’,4’-trihydroxy-4-methoxychalcone (compound 8) using Autodock 4.2.6.

Cpd.	Vdw + Hbond Energy (kcal/mol) [1]	Electrostatic Energy (kcal/mol) [2]	Desolvation Energy (kcal/mol) [3]	Intermolecular Energy (kcal/mol) [4]	Total Internal Energy (kcal/mol) [5]	Torsional Free Energy (kcal/mol) [6]	Unbound System’s Energy (kcal/mol) [7]	Estimated Free Energy of Binding (kcal/mol) [4 + 5+6-7]
7	−8.31	0.17	2.77	−5.36	−0.40	1.79	0.00	−3.97
8	−8.39	0.20	2.70	−5.49	−0.67	2.09	0.00	−4.07
Δ	0.08	0.03	0.07	0.12	0.27	0.30 *	0.00	0.10

The lower energy between the two compounds is highlighted in black, and the asterisk indicates the largest difference between the two chalcones.

## Data Availability

Data sharing is not applicable.

## Sample Availability

Samples of the extracts are available from the authors.
